The article "Motion Fatigue State Detection Based on Neural Networks" was published in 2022. Journal: Comput Intell Neurosci.

# Motion Fatigue State Detection Based on Neural Networks

**DOI:** 10.1155/2022/9602631

**Published:** 2022-03-15

**Authors:** Hu Li, Yabo Wang, Yao Nan

**Affiliations:** Lanzhou City College Sports Institute, Lanzhou 730070, China

## Abstract

Aiming at the problem of fatigue state detection at the back of sports, a cascade deep learning detection system structure is designed, and a convolutional neural network fatigue state detection model based on multiscale pooling is proposed. Firstly, face detection is carried out by a deep learning model MTCNN to extract eye and mouth regions. Aiming at the problem of eye and mouth state representation and recognition, a multiscale pooling model (MSP) based on RESNET  is proposed to train the eye and mouth state. In real-time detection, the state of the eye and mouth region is recognized through the trained convolution neural network model. Finally, the athlete's fatigue is determined based on PERCLOS and the proposed mouth opening and closing frequency (FOM). The experimental results show that in the training process, we set the batch_size = 100 and the initial learning rate = 0.01. When the evaluation index is no longer improved, the learning rate is reduced by 10 times to 0.001, and a total of 50 epochs are trained. The precision and recall of the system are high. Compared with the infrared image simulating the night state, the RGB image taken by the ordinary camera in the daytime has higher precision and recall. It is proven that the neural network has high detection accuracy, meets the real-time requirements, and has high robustness in complex environments.

## 1. Introduction

As shown in Figure 1, machine learning is the general name of a class of algorithms. It automatically analyzes a large amount of data to obtain new knowledge, accumulate experience, make it continuously improve its own performance, and use these laws to identify existing data for prediction or classification. In the fatigue motion detection algorithm based on image processing, machine learning algorithms are mainly used to detect and identify athletes' fatigue states [1]. In the process of fatigue motion detection, some classical machine learning algorithms are used. For example, the AdaBoost algorithm is used to detect the facial region, and then the eye and mouth images are obtained for subsequent processes. Support vector machine (SVM) algorithm is used to classify the manually extracted feature vectors so as to identify the eye state. Using neural network algorithms for face detection and keypoint location, constructing convolution neural network to automatically extract athletes' fatigue features, classify and recognize them, and so on. The other is to automatically extract the fatigue characteristics of athletes by using convolutional neural networks and construct two convolutional neural network models to perform classification tasks for eye and mouth states, respectively, that is, open or closed states [2].

The article "Motion Fatigue State Detection Based on Neural Networks" was published in 2022. Journal: Comput Intell Neurosci.

## 2. Literature Review

Liu Zhiqiang and others proposed a support vector machine (SVM) fatigue detection model based on the ASL eye tracker [3]. Wang Lei and others carried out a 36 h sleep deprivation experiment with an eye tracker to determine the thresholds of three fatigue judgment indicators: PERCLOS value, average eye closing time, and yawning frequency [4]. Nuevo and others used infrared devices to capture the eye movements of moving people and proposed a detection model based on AAM and PCA [5]. Jinjun Wang and others proposed a fatigue detection model based on the hidden Markov method based on simulated mover and infrared imaging [6]. Zeng Youwen and others also used contact instruments to collect physiological information from athletes. In the fatigue exercise experiment, they analyzed the correlation between EEG data and blink times and came to the conclusion that the EEG signal index and the blink time index can maintain the same conclusion when indicating the fatigue degree of athletes. There are also many studies on how to use machine learning methods to analyze EEG signals [7]. Ye Chun and others designed a fatigue detection system for sportspeople based on Morlet wavelet theory and EEG signals, which has the advantages of fast operation speed and strong real-time performance [8]. Xie Zhi and others used the fusion K-means clustering method to process EEG signals. This method can fully consider individual differences and achieve an 80% recognition effect [9]. Kwok Tai Chui and others used the SVM algorithm to process EEG signals. The algorithm has less computation, fast running speed, and an average processing delay of only 0.55 ms [10]. Chin Teng Lin and others used the principal component analysis method to process EEG signals, which has a large amount of calculation and high accuracy [11]. Lee and others made innovations in physiological signal acquisition instruments, using watch-type instruments to collect information such as ECG signals and arm movement status of athletes for fatigue early warning. This acquisition equipment is smaller, easier to popularize, and can ensure that the routine operation of athletes is not affected [12]. Xintong and others used the AdaBoost algorithm for face detection, combined with the prior knowledge such as the geometric proportion of facial features to locate the coordinates of eyes and mouth, finally used the gray-scale integral projection method to extract the opening of eyes and the roundness of mouth as fatigue features, and determined fatigue according to the PERCLOS principle [13]. Wu Minjie and others adopted a similar algorithm design idea, combined with the AdaBoost algorithm and template matching algorithm to complete the function of fatigue feature extraction, and introduced the frequency of mouth opening and closing as one of the criteria into the fatigue detection system of sportspeople [14]. You Feng and others, as shown in Figure 2, after using the AdaBoost algorithm to detect a face, they use an elliptic curve fitting method to obtain eye-opening so as to judge fatigue [15].

The article "Motion Fatigue State Detection Based on Neural Networks" was published in 2022. Journal: Comput Intell Neurosci.

Fatigue detection based on visual image processing has been a research topic for many years. However, due to the large interference of ambient light and human expression in the real scene, the accuracy of face detection and facial behavior feature detection still needs to be improved. To solve this problem, this paper proposes a cascade deep learning structure and a fatigue state detection model based on multiscale pooling networks (MSP net) [16]. The trained MTCNN model is used to detect the face, extract the data of eyes and mouth, put the data of eyes and mouth into the trained MSP net CNN for detection, judge the opening and closing of eyes and mouth, and finally jointly judge fatigue according to PERCLOS and frequency of open mouth (FOM). The specific process is shown in Figure 3.

## 3. Neural Network MSP Net

### 3.1. Pretreatment

#### 3.1.1. Data Acquisition

The fatigue detection system in this paper adopts the cascade form of two deep learning models; one is MTCNN for detecting faces and extracting eye and mouth images, and the other is a multiscale pooled CNN for judging the state of eye and mouth images as proposed in this paper. Both networks require pretraining. Because the deep learning model has made remarkable achievements in face detection in recent years, this paper uses the existing excellent network to obtain the face and eye mouth area and focuses on the fatigue detection task [17]. The MTCNN model used in this paper is a trained model. The author uses the widerface database. There are about 200000 face images, including frame annotation and five key point information (center coordinates of two eyeballs, nose tip coordinates, and two mouth corner coordinates). The regression of network training is the face frame and the coordinates of five key points. The data of eye and mouth image state judgment network training are independently collected by the author in practical work, including some actual athlete images and 21 volunteers. Considering that athletes have night training, the acquisition equipment uses infrared cameras in addition to ordinary cameras. In the process of image and video acquisition, various complex environmental problems of athletes during actual sports are comprehensively considered. The collected image data includes eyes closed, mouth open and closed, no glasses, wearing glasses, front and side, etc. After collection, we filter and eliminate some noise samples. Finally, the selected samples are classified as the opening, closing, opening and closing of ordinary cameras and the opening, closing, opening and closing of infrared cameras. Among them, there are 36764 samples in the eyes and 15185 samples in the mouth [18].

The article "Motion Fatigue State Detection Based on Neural Networks" was published in 2022. Journal: Comput Intell Neurosci.

#### 3.1.2. Data Preprocessing

Because the brightness of the sample image collected by the infrared camera is generally low, the effect of directly putting it into the network training is not good, so the sample needs to be preprocessed. This paper uses the histogram equalization method. The purpose of histogram equalization is to enhance the local contrast. Its main steps are to calculate the cumulative probability of the gray level of the original image and map the original gray value to the new gray value according to the mapping relationship. For example, the gray-scale mapping relationship of gray-scale images with gray-scale values of 0–255 is as follows:

(1) $$\begin{array}{c} p_{k}=255\times \sum_{i=0}^{k}\frac{n_{i}}{n},\;k=0,1,2,\ldots ,L-1, \end{array}$$

where *p*_*k*_ represents the gray value after mapping; *k* represents the kth gray level; *L* gray levels in total; *n* represents the number of all pixels; *n*_*i*_ represents the number of pixels of the i-th gray level; and the resulting *p*_*k*_ is rounded at the end.

### 3.2. Face Detection

Traditional face detection algorithms, such as AdaBoost or frame difference, have poor robustness to complex environments. A deep learning model has great advantages in this regard. In this paper, the MTCNN model is used for face detection. The network structure of MTCNN is mainly divided into the following three layers:

- *P-Net.* Firstly, the image pyramid is constructed, and then the candidate face windows and bounding box reregression vectors are obtained through a fully convolutional network (FCN), which are used to calibrate the candidate face windows. Then, nonmaximum suppression (NMS) is used to merge highly coincident candidate regions [19].
- *R-Net.* We put the candidate areas obtained by p-net into this network to further screen out a large number of wrong candidate areas and perform calibration. Finally, NMS is also used to merge candidate areas.
- *O-Net.* This layer of the network is similar to R-Net, but this layer is made more detailed, and the candidate areas will be more strictly supervised. Finally, five more key point coordinates will be output [19].

The article "Motion Fatigue State Detection Based on Neural Networks" was published in 2022. Journal: Comput Intell Neurosci.

MTCNN has good robustness and can still accurately detect the face rotated at a certain angle. The face is detected by MTCNN, and the eyes and mouth can be successfully marked according to the returned five key points.

### 3.3. Model Design

The multiscale pooled convolutional neural network (MSP net) model is improved on the basis of the structure of RESNET, retains the concept of residual, and modifies the original max pooling to the multiscale pooling (MSP) proposed in this paper at the pooling layer to improve the recognition effect of images collected at different resolutions [20]. The structure of MSP is shown in Figure 4.

The steps of the MSP module are as follows: (a) first passed through twice max pooling to obtain a group of feature maps with side lengths four times smaller than the original feature map. (b) The original feature map is scaled, the side length is doubled, and then the new feature map is max pooled to obtain another group of feature maps with a side length of 1/4 of the original feature map. (c) Scaled the original feature map again, and the side length is reduced to 1/4 times of the original. (d) The three output feature maps are cascaded and introduced into the subsequent deep learning network [21]. The idea of a multiscale pooling model comes from the spatial pyramid pooling model. Compared with the spatial pyramid model, the advantage of multiscale pooling is that its substitution position is more flexible and can be used many times at the beginning, middle, or end of the network.

The structure of the MSP net network designed in this paper is shown in Figure 5. The training methods for the eyes and mouth are the same. Here, we take eyes as an example. In MSP net, the input image is 48 × 48 sizes gray image, after one convolution and MSP output 12 × 12 × 48. The convolution kernel size is 3 × 3. After that, a residual block is passed. There are two layers of convolution in the residual block, and the size of the convolution kernel is still 3 × 3. Residual block output is 12 × 12 × 48 feature maps. After another –max pooling, the output is 6 × 6 × 48 feature maps. Then, the feature maps are converted into a one-dimensional vector and entered into the full connection layer. The input sequence length of the full connection layer is 1728, and there is a hidden layer with a length of 1000. Finally, the classification results are output by Softmax. The categories are divided into four categories: ordinary camera opening, infrared camera opening, ordinary camera closing, and infrared camera closing.

The article "Motion Fatigue State Detection Based on Neural Networks" was published in 2022. Journal: Comput Intell Neurosci.

In order to verify the effectiveness of the MSP net, this paper not only uses the MSP net for experiments but also uses the classical Alex net and RESNET structures as comparison networks for training, testing, and related comparison experiments.

### 3.4. Loss Function and Optimization Method

Finally, the network uses the Softmax classification method, which is divided into four categories. The SoftMax function is defined as follows:

(2) $$\begin{array}{c} p_{j}=\frac{\exp\left(y_{j}^{\prime }\right)}{\sum_{k=0}^{3}\exp\left(y_{k}^{\prime }\right)},\;j=0,1,2,3, \end{array}$$

where *p*_*j*_ represents the probability of class *j*; *y*_*j*_′=∑_*i*_*h*_*i*_*w*_*i*,*j*_+*b*_*j*_ represents the output of the last layer of the full connection layer, *h*_*i*_ is the output of the previous layer, and *w*_*i*,*j*_ and *b*_*j*_ are the weight and offset of the last layer, respectively. The loss function is defined as cross-line and expressed as

(3) $$\begin{array}{c} L_{m}=-\sum_{j=0}^{3}1\left\{y=j\right\}\log\;p_{j}, \end{array}$$

where *L*_*m*_ represents the cross-line of the *m*-th sample; 1{*y*=*j*} represents the indicative function, that is, when *y* = *j*, the function is 1, and when *y* ≠ *j*, the function is 0. (3) is the loss function of a single sample. When there are *M* training samples, the loss function needs to be averaged and it is expressed as

(4) $$\begin{array}{c} L=\frac{1}{M}\sum_{m=1}^{M}L_{m}. \end{array}$$

The optimization method uses adaptive motion estimation (Adam).

### 3.5. Fatigue State Detection

#### 3.5.1. PERCLOS

PERCLOS is the ratio between the number of eye closure frames per unit time and the total number of frames per unit time. The calculation formula is as follows:

(5) $$\begin{array}{c} f_{\text{per}}=\frac{n}{N}\times 100, \end{array}$$

where *n* represents the number of closed eye frames and N represents the total number of frames per unit time. PERCLOS can well quantify the degree of athletes' eye closure. When PERCLOS reaches a certain threshold, it can be judged that the athletes' eye closure time is too long, and it can be preliminarily considered that they have entered a fatigued state.

#### 3.5.2. Mouth Opening and Closing Frequency

FOM, similar to PERCLOS, represents the ratio between the number of frames with mouth open per unit time and the total number of frames per unit time. The calculation formula is as follows:

(6) $$\begin{array}{c} f_{\text{fom}}=\frac{n}{N}\times 100. \end{array}$$

Like PERCLOS, *n* represents the number of shut-up frames and *N* represents the total number of frames per unit time. The greater the value of these two indicators, the greater the degree of fatigue. The final fatigue state detection needs to be considered together.

The article "Motion Fatigue State Detection Based on Neural Networks" was published in 2022. Journal: Comput Intell Neurosci.

#### 3.5.3. Fatigue State Detection

After the pretraining of all deep networks is completed, the threshold of fatigue state is set according to PERCLOS and FOM, and the whole network system is applied to real-time detection. The specific steps are as follows: the camera captures the athlete's video, and MTCNN captures the face and five key points in each frame and extracts the eye and mouth areas. An MSP net is used to detect the state of the eyes and mouth captured in each frame and save them in a fixed long queue. The algorithm detects the change of the median value in the queue in real-time. When the distribution of all values in the queue reaches the threshold fatigue state, the alarm mechanism starts to remind athletes that they have entered fatigue.

## 4. Experimental Results and Analysis

This paper constructs a neural network model based on the deep learning framework and uses the framework of multithreaded input data provided by tensor flow to combine the training data (batch) and disrupt the data order, which can improve the efficiency of model training. During training, we set the batch_ size = 100 and learn_ rate = 0.01. When the evaluation index is no longer improved, the learning rate decreases 10 times to 0.001 and the lowest to 0.00001. One epoch means that all training sets are trained once. In this paper, 50 epochs are trained on the training set, the Adam adaptive moment estimation optimization algorithm is used for backpropagation, the callback function is set to monitor the loss val_loss of the verification set, and the network model with the minimum loss on the verification set is saved as the final training model. The graphs of training loss and verification loss val_loss are shown in Figure 6, and the graphs of accuracy rate train accuracy on training set and accuracy rate val_accuracy on verification set are shown in Figure 7.

The verification dataset and test dataset are used to test the model saved after training. The detection accuracy on each dataset is shown in Table 1.

In order to verify the performance of the algorithm proposed in this paper, using the public CEW dataset, our algorithm is compared with the eye state recognition algorithm proposed in recent years. The detection accuracy is shown in Figure 8.

The algorithms proposed in the above other references collect monocular images to analyze the eye state, while our algorithm analyzes the athlete's eye state through binocular images. Compared with monocular images, the proposed algorithm can extract more abundant features and has higher detection accuracy. The images in the CEW dataset are ideal, and there are few postures such as head deflection and tilt. The experimental results show that our algorithm has high detection accuracy compared with other algorithms. In the yaw DD dataset, the head posture of athletes is changeable, and there will be inclination, deflection, and other situations, where the detection effect of other algorithms will be worse.

The article "Motion Fatigue State Detection Based on Neural Networks" was published in 2022. Journal: Comput Intell Neurosci.

After preparing the training dataset, the next step is to train the network and verify the performance of the network model. This paper uses the framework of multithreaded input data provided by tensor flow to combine training data (batch), which also disrupts the order of training data. In the training process, we set the batch_size = 100 and learn_rate = 0.01. When the evaluation index is no longer improved, the learning rate decreases 10 times to 0.001, and a total of 50 epochs are trained. In this paper, the Adam adaptive optimization algorithm is used for backpropagation, the callback function is used to monitor the loss of the verification set, and the network model with the least loss on the verification set is saved as the final training model. The graphs of training loss train_loss and verification loss val_loss are shown in Figure 9, and the graphs of accuracy on the training set and accuracy val_accuracy on verification set are shown in Figure 10.

The model saved after training is tested with the mouth verification dataset and the test dataset. The detection accuracy on each data set is shown in Figure 11.

In order to verify the performance of the algorithm proposed in this paper, using the public yaw DD dataset, our algorithm is compared with the mouth state recognition algorithm proposed in recent years. The experimental results are shown in Figure 12. Compared with other mouth state recognition algorithms, the algorithm proposed in this paper performs mouth correction, so the detection accuracy is higher when the athlete's head posture is tilted and deflected. Experimental results also show that the proposed algorithm is better than other algorithms.

It can be seen from Figure 13 that videos of athletes under normal exercise, talking/laughing, and yawning are selected from the test dataset. The following two figures are the results of analyzing the fatigue degree of athletes through the state of their mouth. When the system detects that the athlete is yawning (Figure 13), an audible warning is issued to remind the athlete to pay attention.

## 5. Conclusion

In this paper, a cascade deep learning structure and a real-time fatigue detection system based on multiscale pooled convolutional neural networks are designed. Firstly, the athlete's face is detected by MTCNN to extract the key positions of eyes and mouth. Then the eye and mouth images are sent to the multiscale pooled MSP net for the state test, and a fixed-length queue is set. The queue saves the detection results of each frame in unit time, and the fatigue state is judged jointly by PERCLOS and mouth opening and closing frequency (FOM). Experiments show that the proposed algorithm has high detection accuracy, can achieve the effect of real-time detection, and has high robustness in complex environments. The method proposed in this paper will be further transplanted and optimized for the embedded platform.

The article "Motion Fatigue State Detection Based on Neural Networks" was published in 2022. Journal: Comput Intell Neurosci.

## Figures and Tables

**Figure 1:** Technical roadmap of the paper.

**Figure 2:** AdaBoost algorithm detection.

**Figure 3:** Algorithm flow.

**Figure 4:** Multiscale pooling (MSP) module.

**Figure 5:** MSP net structure.

**Figure 6:** Model loss on eye dataset model_loss.

**Figure 7:** Model accuracy on eye dataset model_accuracy.

**Figure 8:** Performance comparison of different eye state detection algorithms.

**Figure 9:** Model loss on dataset model_loss.

**Figure 10:** Model accuracy on mouth dataset model_accuracy.

**Figure 11:** Detection accuracy on each mouth dataset.

**Figure 12:** Performance comparison of different mouth state detection algorithms.

**Figure 13:** Two different mouth states: (a) Normal and (b) Yawning.

**Table 1:** Detection accuracy on each eye dataset.

Dataset	CSW data	Yaw DD data (%)	Self-built data (%)	Average detection accuracy (%)
Validation set	0	98.7	98.6	98.65
Test set	97.87%	98.2	98.44	98.17
Average detection accuracy	97.87%	98.45	98.54	98.42

## Data Availability

The datasets used and/or analyzed during the current study are available from the corresponding author on reasonable request.
